# Clinical and laboratory findings and therapeutic responses in children with nephrotic syndrome

This article has been retracted.

**DOI:** 10.4103/0971-4065.65297

**Published:** 2010-04

**Authors:** A. A. S. L. Safaei, S. Maleknejad

**Affiliations:** Department of Pediatrics, Guilan University of Medical Science, Rasht, IR Iran

**Keywords:** Children, complication, corticosteroid, nephrotic syndrome, pathology

## Abstract

Nephrotic syndrome (NS) is a clinical entity characterized by massive loss of urinary protein leading to hypoproteinemia and edema. This prospective cross sectional study was performed on 44 children with idiopathic nephrotic syndrome (INS). The objectives were to study the clinical and biochemical parameters at the time of diagnosis of nephrotic syndrome and to study the histopathological distribution of different subtypes of INS and drug response pattern. There were 29 (66%) males and 15 females (34%). The mean age of NS was 4.87±3.24 years. Facial edema was found in 42 (95%), microscopic hematuria in 10 (23%), gross hematuria in 2 (4.5%), and hypertension in 5 (11.2%) of patients. In 17 children who underwent biopsy, focal segmental glomerulosclerosis was the most common pathologic finding (41%). Other subtypes included minimal change in three (18%), membranoproliferative glomerulonephritis in 1(5.8%), diffuse proliferative glomerulonephritis in 2 (11.6%), membranous glomerulonephritis in 1 (5.8%), and diffuse mesangial proliferation in 3 (17.5%) of cases. At the time of hospital admission, peritonitis were present in five (11.4%), pneumonia and upper respiratory infection (sinusitis) in eight (18%), cellulitis in two (4.5%). Among 44 children with NS, 29 (66%) were steroid sensitive cases, nine (20.5%) were steroid resistant and six (13.5%) were steroid dependent. Among patients with steroid sensitive NS, 37% were without relapsers, 38.8% frequent relapsers and 26.4% were infrequent relapsers. These results suggest that there are differences between season of incidence, response to treatment with corticosteroid and pathologic findings in our study and other studies in Iran and other countries.

## Introduction

Nephrotic syndrome (NS) is characterized by massive loss of urinary protein (primarily albuminuria) leading to hypoproteinemia (hypoalbuminemia) and its result, edema. Hyperlipidemia, hypercholesterolemia, and increased lipiduria are usually associated. Although not commonly thought of as part of the syndrome, hypertension, hematuria, and azotemia may occur. NS is categorized into primary and secondary forms. The primary NS (PNS) occurs without any previous disease and in some circles, the older designation of idiopathic NS (INS), but both terms denote a similar vagueness as to cause. Included are a variety of clinical as well as pathologic states. The term secondary NS relates to some clinical disease such systemic lupus erythematosus, diabetes mellitus, sickle cell disease or syphilis. Secondary NS is rare in children. The overall prevalence of NS in childhood is approximately 2-5 cases per 100,000 children. The cumulative prevalence rate is approximately 15.5 cases per 100,000[1,2] Minimal change NS is the most common form in children, and its prevalence is inversely proportional to age (i.e., the younger the child, the more likely the histology will show minimal abnormalities on light microscopic evaluation of glomerular histology). Data on differences in racial predilection to NS in children are lacking[1,3–5] in children younger than eight years at onset, the ratio of males to females varies from 2:1 to 3:2.[1,2,5] In older children, adolescents and adults, the male to female prevalence is approximately equal.[4] Histologic variations exist within this category in which some patients demonstrate only fusion and smudging of the epithelial cell podocytes while others may demonstrate mild changes within the glomerular mesangium consisting of either proliferation or sclerosis. Since patients with minimal change NS have the highest rate of responsiveness to standard treatment and best long-term prognosis, the separation of minimal change NS from others is important.[6–8]

## Materials and Methods

This prospective cross sectional study was performed on 44 children with idiopathic NS, in 17 Shahrivar hospital (with age at onset up to 14 years) Most patients were referred to our unit for further management. All patients fulfilled the International Study of Kidney Disease in Children (ISKDC) criteria, for the diagnosis of nephrotic syndrome: urinary spot protein/creatinine >2.0, serum albumin <2.5 g/dl, serum cholesterol >200 mg/dl, and edema.[1] The study parameters included age, sex, nationality, presenting symptoms and blood pressure of the patients, complete blood picture, urine analysis and microscopy, 24-hour urinary protein excretion, creatinine clearance, serum electrolytes, serum urea and creatinine levels, serology and immunological studies, serological markers for hepatitis B and C, antibody against the human immunodeficiency virus (HIV), ultrasound, treatment and outcome.

After informed consent, kidney biopsy was performed in the following situations:

1. age at onset less than one year and more than than 10 years,
2. no response to eight weeks of prednisolone therapy,
3. frequent relapser (FR), steroid-dependent (SD), and steroid non-responder (SNR) categories and before cyclosporine therapy, and
4. unusual clinical features (hypertension and micrscopic hematuria) and/or laboratory abnormalities (abnormal renal function and low c3 and c4).[1,2,4]

The biopsy specimens were evaluated histopathologically by light and immunofluorescence microscopy. An adequate biopsy was defined as the presence of at least 10 glomeruli in the specimen on light microscopy.

The response to treatment was classified according to the definitions from ISKDC: (a) steroid sensitive–complete resolution of proteinuria within eight weeks of prednisone therapy; (b) steroid resistance–failure to respond to eight consecutive weeks of treatment with prednisone at 2 mg/kg/day; (c) steroid dependence–recurrence of nephrosis when the dose of corticosteroids is reduced or within two months after the discontinuation of therapy; (d) frequent relapsers–two or more episodes of nephrosis within six months of the initial response or four or more within any 12-month period (not related to changes in prednisone dose)[1,2] steroid dependent patients, frequent relapsers, steroid resistant patients candidates for alternative agents, particularly, levamisol, cyclophosphamide, cyclosporine, mycofenolate mofetil and tacrolimus.[1,9,10] We obtained data regarding age, sex, and presenting features, laboratory finding, response to treatment and biopsy results using a standardized data–sheath.

## Results

There were 29 males (66%) and 15 females (34%); male to female ratio was 1.9/1. The mean of idiopathic NS was 4.87±3.24 years (range of neonate to 14 years). One of these patients had congenital NS. Fifteen patients were admitted to the hospital in spring (34.1%) and other patients were admitted in winter (18.2%), summer (25%) and fall (22.7%). The mean level of serum albumin was 1.75±0.45 g/l, The mean level of 24-hour urinary protein excretion 3344.84±2344.38 mg/dl, mean level serum cholesterol was 473±160 mg/dl and mean serum of triglyceride was 335.4±113.8 mg/dl. The most common presenting signs and symptoms were facial edema in 42 (95%), limb edema 36 (82.2%), scrotal edema 24 (54.5%) anasarca in 18 patient (41%) abdominal pain in eight (18.2%), diarrhea in four (9%) ascitis in 28 (64%) pleurisy in four (9%), anorexia in 24 (54.5%), hypertension in 5 (11.2%) microscopic hematuria in 10 (23%) and gross hematuria in two patients (4.6%). All patients of the studied group were seronegative for HBsAg and HIV. Evaluation for complication of disease was done in all patients. Acute renal failure due to low serum albumin and overenthusiastic diuretic consumption in other centers were seen in eight patients (18%). Acute renal failure was seen in seven patients and renal biopsy was done in one patient because of persistent acute renal failure, and renal pathology was compatible with focal segmental glomerolusclerosis. Regarding hospital admission, peritonitis were present in five (11.4%), pneumonia and upper respiratory infection in eight (18%) and cellulitis in two (4.5%) patients. In follow-up, primary disease progressed toward end stage renal disease (ESRD) in four (9%) patients. Ultimately, renal transplantation was performed in two cases with FSGS. Detail of age and sex distribution of patients are shown in [Table 1].

**Table 1:** Age and sex distribution of 44 patients with NS

Age (Years)/Sex	Male	Female	Percent	Total
<1	1	-	2.2	1
1-5	19	12	70	31
6-10	6	12	18.8	8
>10	3	1	9	4

Kidney biopsy was performed in 17 (38.4%) of 44 patients. FSGS was the most common histopathological subtype in seven of 17 children (41%), Other subtypes included minimal change disease in three (18%), membranoproliferative glomerulonephritis (MPGN) in one (5.8%), diffuse proliferative glomerulonephritis in two (11.6%), membranous glomerulonephritis in one (5.8%), and diffuse mesangial proliferation in three (17.5%). Among 44 children with NS, 29 cases (66%) were steroid sensitive, nine (20.5%) were steroid resistant and six (13.5%) steroid dependent. Of patients with steroid sensitive nephrotic syndrome, 37% were non-relapsers, 38.8% frequent relapsers and 26.4% infrequent relapsers. Among those with steroid resistant NS, seven had focal segmental glomerulosclerosis and 2 had DMP. In this study only one patient with FSGS died because of end stage renal disease.

## Discussion

In this study, we analyzed all children with INS who referred to 17 Sharivar Hospital. In our study the male to female ratio was 1.9/1. According to two studies in Turkey, male to female ratio was 1.6/1 and 1.7/1 (6, 7). According to a study in India carried out by Kumar *et al*. male to female ratio was 2.76/1.[11]

A study by Madani *et al*. on 502 patients in Center Medical Pediatric showed that 63.7% were male and 36.3% female with a male to female ratio 1.75/1.[8] In the report which was presented by Sorkhi in Babol hospital, male to female ratio was 1.6/1.[12] Considering these results, it can be said that differences in sex predilection to NS and maybe even a more pronounced difference in the types of NS acquired within a geographic area exist although in all of studies male involvement was more. In our report, 31 cases of patients were in the age range 1-5 years (71%). Only one patient had congenital NS, admitted at age 45 days. In this study the mean age of patients at onset of INS was 4.87±3.24 years (range neonate to 14 years). In a study by Kumar *et al*. in India, the mean age of patients at the onset of NS was 7.9±5.1 years[11]; other studies in New Zealand and and Saudi Arabia showed that the mean age was 5.4±3.9 and 4.3±3.1.[13,14] According to a report from Center Medical Pediatric by Madani *et al*.[8] 337 cases of 502 patients were in the range of 1-5 years (67%). Another study by Sorkhi *et al*., performed on 75 children, showed that 62.5% patients were in the range of 2-8 years.[12] These results suggest there are difference in age distribution of patients but our findings are relatively similar to results obtained in the two centers in Iran.

In this study, 15 patients were admitted to the hospital in spring season (34.1%), other patients were admitted in winter (18.2%), summer (25%) and (22.7%) in fall. However, according to a report by Sorkhi *et al*. 38% of cases admitted in winter differed from our results;[12] the most common presenting signs and symptoms were facial edema in 42 (95%), limb edema 36 (82.2%), scrotal edema 24 (54.5%) anasarca in 18 patient (41%) abdominal pain in eight (18.2%), diarrhea in four (9%) ascitis in 28(64%) pleurisy in four(9%) anorexia in 24(54.5%) hypertension in 5(11.2%) microscopic hematuria in one (23%) and gross hematuria in two (4.6%) patients.

The presenting signs and symptoms in our study, differed from others; for example, frequency of microscopic hematuria and hypertension in Indian children was 41 and 26.8% respectively.[9,14] FSGS was the most common histopathological subtype in seven of 17 children (41%). Other subtypes included minimal change disease in three (18%), membranoproliferative glomerulonephritis (MPGN) in one (5.8%), diffuse proliferative glomerulonephritis in two (11.8%), membranous glomerulonephritis in one (5.8%), and diffuse mesangial proliferation in two (11.8%) and focal and segmental endocapilary proliferation in one patient (5.8%).

Results of renal biopsy in 138 Turkish children showed that in 49% of cases pathologic findings were compatible with mesangial proliferate glomerulonephritis.[6,7] Another study carried out Kumar *et al*. in India showed that FSGS was the most common histopathological subtype in 110 of 387 children with NS (38%). According to the Madani *et al*. study, minimal change disease was the most common histopathological subtype in 67(34/4%) children.[8] This study, in comparison with other studies in other countries and centers, showed variable histology pattern, although at this time it is seems that minimal change disease is the most common variation of nephrotic syndrome in children. These differences may be related to racial, genetic and environmental factors.[3,6,11,13,15–16] Among 44 children with NS, 29 cases (66%) were steroid sensitive and 9(20.5%) steroid resistant and six (13.5%) were steroid dependent. Among patients with steroid sensitive NS, 37% were non-relapsers, 38.8% frequent relapsers and 26.4% infrequent relapsers. Among those with steroid resistant NS seven cases had focal segmental glomerulosclerosis and 2 had DMP.

Other studies have shown that corticosteroid sensitivity in patients is variable:[17,18] in Ozkaya report 76%,[6] Madani 79.2%,[8] Ahmadzadeh 87%,[19] Srivastava 77%,[20] Asinobi 78%.[10]

In our study, two patients died - one of them due to congenital NS and the other because of complicatons due to end stage renal disease.

## Conclusion

This study suggests there are differences in incidence, responses to treatment with corticosteroid and pathology findings of biopsy among studies conducted in Iran and other countries.

## References

[1] Niaudet P, Avner ED, Harmon WE, Niaudet P (2004). Steroid-sensitive idiopathic nephrotic syndrome. Pediatric Nephrology.

[2] Burgstein JM, Behrman RE, Kliegman RM, Jenson HB (2008). Nephrotic syndrome. Nelson Textbook of Pediatrics.

[3] Churg J, Habib R, White R (1970). Pathology of the nephrotic symdrome in children.A report from the International Study of Kidney Disease in children. Lancet.

[4] Falk JR, Jennette JC, Nachman PH, Brenner BM, Levine SA (2004). Primary glomerular disease. The Kidney.

[5] Hawkins P, Millan JA, Angelis CD, Feigin RD (2000). Nephrotic Syndrome. Oski pediatrics principles and practice.

[6] Ozkaya N, Cakar N, Ekim M, Kara N, Akkok N, Yalcinkaya F (2004). Primary nephrotic syndrome during childhood in Turkey. Pediatr Int.

[7] Bircan Z, Yilmaz AY, Katar S, Yildrim M (2002). Childhood idiopathic nephotic syndrome in turkey. Pediatric Int.

[8] Madani AB (2003). Clinicopathologic and drug response in children with idiopathic nephrotic syndrome in pediatric medical center. J Tehran University Med Sci.

[9] Bayazit AK, Noyan A, Cengiz N, Anarat A (2004). Mycophenolate Mofetil in the children with Multidrug-resistant nephrotic syndrome. Clin Nephrol.

[10] Asinobi AO, Gbadegesin RA, Ogunkunle OO (2005). Increased steroid responsiveness of young children with nephrotic syndrome in Nigeria. Ann Trop Pediatr.

[11] Kumar J, Gulati S, Sharma AP, Sharma RK, Gupta RK (2003). Histopathologial spectrum of childhood nephrotic syndrome in Indian children. Pedatr Nephrol.

[12] Sorkhi HA (2002). Steroid response in children with nephrotic syndrome in amirkola hospital. J Babol University Med Sci.

[13] Kari JA (2002). Changing trends of histiopathology in childhood nephrotic syndrome in western Saudi Arabia. Saudi Med J.

[14] Simpson AK, Wong W, Morris MC (1998). Pediatric nephrotic syndrome in Auckland, New Zealand. J Ped.

[15] Craing GC, Willis NC, Hodson EM (2000). Incidence of nephrotic syndrome in children in Australia. Ped Nephrol.

[16] Filler G (2003). Treatment of nephrotic syndrome in children and controlled trials. Nephrol Dial Transplant.

[17] (1981). International Study of Kidney Disease in Children: Primary nephrotic syndrome in children: clinical significance of histopathologic variants of minimal change and of diffuses mesangial hypercellularity. A Report of the International Study of Kidney Disease in Children. Kidney Int.

[18] Vehaskari VM (2005). High incidence of initial and late steroid resistance in childhood nephrotic syndrome. Kidney Int.

[19] Ahmadzzadeh A, Derakhshan A (2007). Idiopathic nephrotic Syndrome in Iran. Indian Ped.

[20] Srivastava RN, Mayekar G, Anand R (1975). Nephrotic syndrome in children. Arch Dis Child.

